# Osteoblastic Cell Responses of Copper Nanoparticle Coatings on Ti-6Al-7Nb Alloy Using Electrophoretic Deposition Method

**DOI:** 10.1155/2022/3675703

**Published:** 2022-04-19

**Authors:** Hanan Ali Hameed, Haider Ali Hasan, Norhayati Luddin, Adam Husein, Azirrawani Ariffin, Mohammad Khursheed Alam

**Affiliations:** ^1^Prosthdontic Department, College of Dentistry, University of Babylon, Iraq; ^2^Oral and Maxillofacial Surgery Department, College of Dentistry, University of Babylon, Iraq; ^3^Prosthodontic Unit, School of Dental Sciences, Universiti Sains Malaysia, Kota Bharu, Kelantan, Malaysia; ^4^Department of Preventive Dental Science, College of Dentistry, Jouf University, Sakaka, Aljouf, Saudi Arabia; ^5^Center for Transdisciplinary Research (CFTR), Saveetha Dental College, Saveetha Institute of Medical and Technical Sciences, Saveetha University, Chennai, India; ^6^Department of Public Health, Faculty of Allied Health Sciences, Daffodil International University, Dhaka, Bangladesh

## Abstract

**Aim:**

To investigate and compare the cell cytotoxicity, proliferation, cell attachment, and morphology of human fetal osteoblasts (hFOB) cells of coated samples (titanium nanocopper (Ti Cu), titanium nanohydroxyapatite (Ti HA) and titanium nanocopper ion doped hydroxyapatite (Ti Cu/HA) and uncoated samples (Ti) in order to assess the suitability of these surface modifications on Ti-6Al-7Nb for dental implant application.

**Materials and Methods:**

The cytotoxicity was studied by examining the hFOB cell response by MTT assessment. The cell morphology was evaluated by inverted microscopy and observed under scanning electronic microscopy (SEM).

**Results:**

MTT assay results displayed that the Cu content on the surface of Ti-6Al-7Nb alloys did not produce any cytotoxic effect on cell viability. The cell viability rate in all samples ranges from 97% to 126%, indicating that hFOB cells grew at a high proliferation rate. However, no significant differences in cell viability were observed between Ti and Ti Cu and between Ti HA and Ti Cu/HA groups. Microscopic examination demonstrated no difference in the cell morphology of hFOB among all samples. In addition, SEM observation indicated favorable adhesion and spreading of the cells on the coated and uncoated samples.

**Conclusions:**

The surface modification of Ti-6Al-7Nb alloy with Cu, HA, and Cu/HA exhibits good cell biocompatibility, and the Cu has no influence on the cell proliferation and differentiation of hFOB.

## 1. Introduction

Replacing missing teeth without affecting the rest of the dentition, while imitating the physiology of a sound tooth for everyday function with good aesthetic appearance, is one of the goals in dentistry. One of the very popular treatment options towards the realization of this dream is dental implants. Commercially pure titanium (Cp-Ti) is among the most widely used as dental implant material because of its biocompatibility and corrosion resistance [1]. Titanium 6-aluminium 7-niobium (Ti-6Al-7Nb) alloy was introduced as a material of choice in dental applications because its mechanical strength was superior to that of Cp-Ti. It is also highly resistant to corrosion and wear [2–4]. Additionally, short-term implantation *in vivo* produced an exceedingly transient inflammatory response to Ti-6Al-7Nb that closely resembled the response to Cp-Ti. No obvious unfavorable biological effects have been reported for both. These results suggested that Ti-6Al-7Nb has favorable biocompatibility and are considered as a promising material for oral implantology. Although biocompatibility and mechanical properties of any biomaterial are among the primary issues for the choice of an implant material, still the success of dental implants is mainly reliant on bone implant osseointegration. Ti-6Al-7Nb still has shortcoming in some properties such as bioinertness which result in poor or inadequate adhesion between bone-implant contact [5, 6]. To reinforce this bone-bonding mechanism, implants have been coated with osteoconductive biomaterials such as hydroxyapatite (HA). This is due to the fact that it possesses similar chemical, structural, and biological properties to that of the human bone, which in turn promotes osseointegration [7, 8]. However, the use of HA has a few drawbacks such as its brittleness in nature limits its use in load-bearing clinical applications. Other than that, the rough surface of HA and absence of antibacterial properties in its component induced an increased risk of bacterial adherence and colonization of metallic implants coated with HA [9].

Bacterial infection is considered as one of the rising complications after implant placement [10, 11]. The recurrent incidence of this infection and repeated use of antibiotics to fight against infection could also lead to the incidence of antibiotic-resistant bacteria. So, the risk for implant failure becomes higher and could bring significant economic burden to the patients and society [12]. As such, introduction of antibacterial agents into HA coating has achieved some growing attention. In recent years, incorporation of metallic antibacterial agents such as copper (Cu^2+^), silver (Ag^+^), and zinc (Zn^2+^) in bioceramics is implemented to aid in the inhibiting microbial growth at the implant site [13–15]. Numerous research reported that the coated implant with metallic ions has a role in minimizing or preventing preliminary bacterial colonization [16–18]. Unfortunately, applications of the inorganic antibacterial agents carrying silver have been avoided due to discoloration issues and high cost. Meanwhile, Cu has becoming a material of growing interest for antibacterial application as it is an essential trace element for mammals to stimulate the activity of several enzymes and performs a function in cross-linking of collagen and elastin of bones. In addition, Cu has been demonstrated to exert high antibacterial ability with low cytotoxicity [13, 19]. Therefore, copper represents a greater promise coating because of its decrease toxicity and good biocompatibility [15]. Despite the fact that higher content of Cu in biomaterials provides better antibacterial effect, the increase of Cu ion might increase the biomaterial cytotoxicity by affecting the cell growth and proliferation [20]. Potential applications of metallic antibacterial agents in dentistry require that agents interact well with oral tissues, in order to produce a sustained antibacterial effect on the time [21]. Additionally, Cu not only influences the antibacterial properties but also influences the mechanical properties such as hardness, rigidity, high yield strength, flexibility, and ductility [22].

The biocompatibility of implant material is a critical issue because this material is in intimate contact with oral tissues for long terms and cannot be removed by the patient. For this reason, the investigation of biocompatibility of any materials used in dental implants is necessary to be carried out to ensure the safety of the material before being used. The most widely used biological systems for *in vitro* toxicity testing of dental materials are cells in culture. Different assays can be used to assess the effects of a biomaterial on cell number, cell growth, cell membrane integrity, enzyme activity, or genetic effects. In addition, cell adhesion and spreading has been suggested as an evaluation criterion. Therefore, *in vitro* biocompatibility tests using MTT assay, light microscopic evaluation, and cell attachment were employed to assess the cytotoxicity of Cu with hFOB cells. Human fetal osteoblast cells were used to evaluate the toxicity of nCu. Up to the best of our knowledge, there is no information about the human fetal osteoblast cell proliferation, morphology, and adhesion associated with Ti-6Al-7Nb alloy coated with copper, hydroxyapatite, and copper ion-doped hydroxyapatite using electrophoretic deposition. Electrophoretic deposition technique offers many advantages that can be used as one of the method to prepare bioceramic coatings on metallic substrates [23–25].

## 2. Materials and Methods

### 2.1. Preparation of Samples

Ti-6Al-7Nb alloy in rod with a diameter of 10 mm was cut into 2 mm in thickness. All samples were ground with silicon carbide abrasive papers up to 2000 grits, polished with 1 *μ*m diamond paste and ultrasonically cleaned with acetone and distilled water. The total samples were divided into 4 groups. The uncoated group acts as a control group (Ti), and other three groups were coated with copper nanoparticles (Ti Cu), hydroxyapatite nanoparticles (Ti HA), and copper ion doped hydroxyapatite nanoparticles (Ti Cu/HA). This study was carried out on three replicate samples for each group. The coating of samples was done by electrophoretic deposition process [26, 27]. Before testing, all samples were sterilized by autoclaving at 121°C for 20 mins.

### 2.2. Cell Culture

#### 2.2.1. Cell Revival and Subculture

Human osteoblast cell lines, hFOB 1.19 (CRL-11372), were purchased from American Type Cell Culture (ATCC) (Manassas, USA). The hFOB cells were cultured in Dulbecco's Modified Eagle Medium F-12 (DMEM/F12) (Invitrogen GmBH, Germany) which was supplemented with 10% fetal bovine serum (FBS) (Invitrogen GmBH, Germany) and 1% penicillin/streptomycin (Invitrogen GmBH, Germany). The cells were incubated in a 5% CO_2_ 37°C humidified incubator (Sheldon, United States) and monitored closely for 24 hours. The aseptic work was maintained by using a laminar flow (ESC II Series, Germany) to avoid contamination of the cultured cells. The laminar flow was sterilized by switching on the ultraviolet (UV) (40 watt) germicidal tubes prior to work.

#### 2.2.2. Cell Viability Assay

According to the International Standard ISO 10993-12 [28], Ti Cu, Ti HA, Ti Cu/HA, and Ti samples were immersed in DMEM/F12 solution with a surface area-to-volume ratio of 1.25 cm^2^/mL. The immersed samples kept under a condition of 37°C and 5% CO_2_ in air for 72 hours to prepare extracts. Cell viability was determined with the 3-(4,5-dimethylthiazol-2yl)-2,5 diphenyl tetrazolium bromide (MTT) according to the manufacturer's protocol. DMEM/F12 medium was used as a blank control sample. The cells were plated at 5 × 10^3^ cells/well with a 100 *μ*L culture medium per well in the 96-well microtiter plate and cultivated at 37 ± 1°C with 5% CO_2_ in air for 24 h. After that, the culture medium was discarded, and then, 150 *μ*L of the extract for testing groups or DMEM/F12 medium for control was added into the wells. The plate was then cultivated at 37 ± 1°C with 5% CO_2_ in air for 1 day and 3 days. After each period of incubation, the culture medium was discarded and 30 *μ*L of MTT stock solution was added into each well, and each plate was incubated for 3–4 h. Subsequently, all the content of each well was changed by 100 *μ*L of dimethyl sulfoxide (DMSO). By using spectrophotometer enzyme-linked immunosorbent assay (ELISA), the optical density (OD) of the solution was measured at a test wavelength of 570 nm (reference wavelength was 600 nm). The statistical significance of differences for treatment groups at day 1 and day 3 was determined using one-way analysis of variance (ANOVA). For the cell viability comparison of the four groups between day 1 and day 3, two-way analysis of variance (ANOVA) was used. The results with *p* value < 0.05 were considered statistically significant.

#### 2.2.3. Cell Morphology

The cell morphology of hFOB was observed using an inverted microscope, Leica DM IL (Wetzlar, Germany). The flask containing the cells was obtained from the incubator and placed on the microscope stage and focused at 4x magnification. For a closer or larger view of the cells, the magnification was changed to 10x, 22x, 40x, and 100x.

#### 2.2.4. Cell Attachment

The cell attachment properties were examined as described by Ahmed et al. [29]. The titanium alloy samples were sterilized using autoclaved and UV in 6-well plates. After preparing the medium having 10^5^ cells, 250 *μ*L of prepared medium was added onto the top of every sample and left for 30 min. After that, at the side of each well, 5 mL of prepared medium was added slowly, and the plate was incubated at 37°C and 5% CO_2_ for 24 and 72 hours. The samples were washed by sterile distilled water after each time interval. Next, 2.5% glutaraldehyde (Merck, Germany) was added for 2 hours, and the samples were dehydrated in ethanol at five concentrations (30% and 50%, 10 min each; 70%, 90%, and 100%, 5 min each) and the samples were dried. After complete dryness, the samples were fitted onto aluminum stubs via carbon double-sided tape, coated with gold using a sputter coating machine (Leica EM SCD005, Czech Republic), and then viewed under scanning electron microscopy (SEM).

## 3. Results

### 3.1. Cell Viability Assay

The cell number was compared among Ti, Ti Cu, Ti HA, and Ti Cu/HA extract after 1 and 3 days of incubation.  Figure 1 shows the OD values for the MTT test after day 1 and day 3 of incubation with the extracts.  Figure 2 shows the cell viability rate of cells on different samples and at different cultivation durations. At day 1, the cell viability rate for Ti HA and Ti Cu/HA is kept at high value larger than 100%, indicating that hFOB cells grew at a high proliferation rate than those on other samples. At day 3, the cell viability rate in all samples was still at high values, and 97%–141% demonstrated that the cells were still with good growth state, but the cell viability rate in Ti samples was significantly lower than in other samples. However, no significant difference in cell viability rate values was observed between Ti and Ti Cu and between Ti HA and Ti Cu/HA at day 1 and day 3 (*p* > 0.05) (Figure 1 and Table 1). According to the cytotoxicity profile of the materials classified by Zhang et al. [30], the results indicate that four groups exhibit no cytotoxicity to hFOB cells and the maximum cell proliferation occurred for Ti HA and Ti Cu/HA. The comparison of cell viability of four groups between day 1 and day 3 presented no significant differences except for Ti Cu/HA.

### 3.2. Morphology of Cells

The morphology of hFOB cells cultivated with DMEM/F12, Ti, Ti Cu, Ti HA, and Ti Cu/HA extract at day 1 and day 3 is shown in Figures 3 and 4, respectively. There was no difference in the cell morphology among the five groups which show that Ti, Ti Cu, Ti HA, and Ti Cu/HA did not bring any variation to the morphology after cultivation. The density of cells that were incubated with DMEM/F12 and extract of Ti HA and Ti Cu/HA was higher than those incubated with Ti and Ti Cu. The cells preserved the typical morphology of hFOB cells from elongated to polygonal appearance with spindle-shaped cells. Furthermore, the cells appeared more confluent at day 3 when compared with day 1.

### 3.3. Cell Attachment

At day 1, all the cells on all surfaces were rounded with raised nuclear regions indicating delayed spreading (Figure 5). After 3 days, the cells became flat and spread, spreading the cells indicating better adhesion on the substrate. The cell attachment to the samples showed that prominent cytoplasmic processes forming more bridges and borders of adjoining cells were fused (Figure 6). The cell proliferation on HA and Ti Cu/HA is better than the other two substrates. The bridges that were formed help cells to cross grooves and spread over them, leading to larger numbers of cells. These results are in agreement with those from MTT assay and light microscopic investigations.

## 4. Discussion

### 4.1. Cytotoxicity

Cytotoxicity measurements on materials used in dental and medical implantology are extremely important. The cytotoxic effect of copper has been evaluated on some substrate and different cells, and favorable results were obtained as suitable antibacterial material for implantology. Nevertheless, it was essential in the current study to evaluate its cytotoxic effect as a coating on Ti-6Al-7Nb alloy by electrophoretic deposition method on hFOB cells. The human osteoblast cell line hFOB 1.19 was used in experiment for the cell culture. These cells showed minimal chromosome abnormalities and synthesize a normal spectrum of matrix proteins [31].

Our results showed that the extracts obtained by Ti, Ti Cu, Ti HA, and Ti Cu/HA samples have no cytotoxic effect on hFOB cells. The Ti Cu/HA revealed significantly superior cell viability than the Ti and Ti Cu and not significantly different compared with Ti HA. This meant that the presence of Cu in the Ti Cu/HA might play effective role in stimulating the growth of cells because the release of Cu may support cell viability and the presence of Cu may change the surface potential to improve cell attachment. Ai et al. [32] showed that the copper element in the HA lattice will be released slowly with the degradation of HA, which can provide low concentration of copper element for a long time and play a role of long-term sterilization and promote the growth of bone cells.

The cell viability rate of coated and uncoated sample extract on hFOB cells after day 3 was nonsignificantly different when compared to day 1 except for Ti Cu/HA group which showed significantly higher cell viability rate. Ewald et al. [33] showed that the cell activity and proliferation of osteoblast on calcium phosphate was improved and the expression of several special osteogenic proteins such as sialoprotein or osteocalcin was affected by copper ion (Cu^2+^). Therefore, the calcium phosphate cement modification with Cu may present a likely alternative to protein-based modification to enhance cell viability for superior bone healing [20]. In addition, copper is an important trace element for human body, and it takes part in many metabolic processes in most of the living organisms [34, 35]. Meanwhile, Cu ions can improve bone healing and enhance vascularization [36, 37]. More importantly, for the soft tissue, copper can be mobilized to the injured sites to increase the host defense and accelerate the healing of early skin wound [38, 39].

Cu shows high antibacterial ability but keeps a low cytotoxicity property. However, better antibacterial effect was provided by higher Cu content in the biomaterials, but at the same time, cytotoxicity was increased [20]. Additionally, the requirements for copper are increased during pregnancy and lactation, and hence, it is critical for growth and development of the fetus and neonate [40, 41]. Moreover, the calcium ions in HA coatings were reported to form sites of positive charges which aid in the adsorption of vitronectin and fibronectin which are the main two proteins that affect cell attachment and spreading [42, 43].

These results in the present study correlated well with Huang et al. [44] who found that the electroplated copper-doped carbonated HA (CuHA) coating on titanium (Ti) had no cytotoxic effect on MC3T3-E1 osteoblast-like cells. Again, the results of current cytotoxicity test are in agreement with Ren et al. [12] who revealed that there was no significant difference in cell viability between Ti-6Al-4V and Ti-6Al-4V-3Cu alloys during the tested period of 2, 4, and 7 days, indicating that the Ti-6Al-4V-3Cu alloy had no cytotoxic effect on L929 cells. Other than that, Zhang et al. [45] found that the different Cu contents in Ti–Cu-sintered alloys exhibited very good cell biocompatibility like Cp-Ti. An increase in the Cu content in the Ti–Cu alloys does not influence the cell viability, cell morphology, and cell differentiation of MG63 cell line. Additionally, Chai et al. [46] observed no difference in the number of MG63 osteoblast-like cells with stainless steel 317L-Cu alloy when compared to Ti-6Al-4V and stainless steel 317L. Also, in Sobierajska et al.'s work [47], nanohydroxyapatites (nHAp) doped with copper and/or zinc ions were investigated for the assessment of its biocompatibility. Three forms of material with diverse surfaces were tested: nanopowder in colloidal suspension, galactose hydrogel (3,6-anhydro-*α*-l-galacto-*β*-d-galactan) scaffold, and pellet. The cytotoxicity evaluation of tested biomaterials showed biocompatible properties of both nanomaterial colloidal solutions as well as galactose hydrogel eluates toward normal mouse osteoblast cell lines (7F2) and human chondrocytes (TC28A2) and osteosarcoma cell line (U2OS). Furthermore, in other study, it was found that if the molar concentration is below the critical point, Cu^2+^ has beneficial effect by improving cell activity and proliferation of osteoblast cells and may also influence osteogenesis protein expression [33, 48].

### 4.2. Light Microscopic Investigations

The histological evaluation of the morphological changes of the hFOB 1.19 cells before and after treatment with the Ti, Ti Cu, Ti HA, and Ti Cu/HA extract was carried out using an inverted microscope to support biochemical evidence. The data of our biochemical seemed to be consistent with the morphological study. The morphological characteristics differ according to cells types. Having spindle and elongated shapes with only slight areas of spreading at the end of long lamellipodia is the most important morphological characteristic of osteoblasts [49]. Figures 3 and 4 show the morphology of hFOB cells cultivated with *α*-MEM, Ti, Ti Cu, Ti HA, and Ti Cu/HA extract for day 1 and day 3, respectively. It showed that all cells maintained the spindle shape and no difference could be found between the samples. These results clearly indicate that from the point of cell morphology, all samples show good cell biocompatibility. This result is supported by Zhang et al. [45] who detected a confluent layer of MG63 cells on the surfaces of both the Cp-Ti and the sintered Ti-10 wt% Cu (Ti–Cu) samples, and no difference can be found in the cell morphology between them. This demonstrates that the Ti–Cu samples did not change the cell morphology during cultivation. Similarly, Sun et al. [50] reported that there are no significant differences in MC3T3-E1 mouse cell morphology between the use of 317L stainless steel with 317L-Cu stainless steel. Based on the results, it was suggested that both types of stainless steel did not initiate cytotoxicity to the mouse cells.

In Sobierajska et al.'s work [47], nanohydroxyapatites (nHAp) doped with copper and/or zinc ions were investigated for the assessment of its biocompatibility. Three forms of material with diverse surfaces were tested: nanopowder in colloidal suspension, galactose hydrogel (3,6-anhydro-*α*-l-galacto-*β*-d-galactan) scaffold, and pellet. The red blood cell morphology evaluation of tested biomaterials showed that unaltered red blood cell morphology was visible after a short and long time of incubation with the obtained biomaterials by using confocal laser scanning microscopy (CLSM). The comparison research provided data of 7F2, TC28, and U2OS cell attachment to the galactose hydrogel surface.

### 4.3. Cell Attachment

The interaction and contact between cells and surface of biomaterial are an important physiological process. In the present study, SEM was used to examine cellular reactions to the alloys by studying hFOB cell morphology on the Ti, Ti Cu, Ti HA, and Ti Cu/HA as shown in Figures 5 and 6. It was shown that the cells on all surfaces were rounded with raised nuclear regions indicating delayed spreading. After 3 days, the cells became flatten and spread, which indicate better adhesion on the substrate. Also, after 3 days of culture, the cells form more bridges on Ti HA and Ti Cu/HA compared to the other two substrates. The bridges formed help the cells to cross grooves and spread over them, leading to larger numbers of cells and thus leading to better cell proliferation. The morphologies demonstrated the absence of a toxic nature for the cells.

It was reported that the response of cells on biomaterials includes the subsequent steps: the adsorption of serum proteins on the specimen, connection of rounded cells on the specimen, and the attachment and spreading of cells to the specimen. In the attachment step, physicochemical connections are implicated between cells and material surface by ionic and/or van der Walls forces [51].

The findings showed well spreading of cells onto all the samples and there proposed good cell viability on the Ti HA and Ti Cu/HA. The cell viability of Ti Cu/HA presented similarity in the morphology of cells to the HA which affirms that Cu does not display any toxic nature. For that reason, it could be concluded that the cell morphology of hFOB cells was not affected with the use of coating Cu. Copper is a fundamental trace element which is necessary to the health of humans, animals, plants, and microorganisms. However, similar to all fundamental elements and nutrients, so much or so little ingestion of copper can result in an identical case of excess or deficiency of copper in the body, each of which can lead to tissue injury and disease [52]. These could explain the higher cell attachment and proliferation viewed on the samples coated with HA. Our result is in agreement with Rad et al. [53] who demonstrated that the number of attached and proliferated MG63 cells on the sample coated with HA using electrophoretic deposition process at dynamic voltage was higher compared to the noncoated titanium sample and culture plate used as control.

In addition, the result of current study is in agreement with Li et al. [54] who reported that the cells appeared round on all HA samples with different roughness at day 1. Meanwhile, the cells become flat and spread at day 3 with little noticeable difference among the samples. In addition, Ren et al. [12] found that there was no obvious difference in cell morphology of L929 cells after coculturing with the extract of Cu wt 3% alloy and Ti-6Al-4V. The cells looked normal and lived in good state on Ti-6Al-4V-3Cu alloy.

## 5. Conclusions

Based on the results of the present study, the following conclusions can be drawn:

1. The cytotoxic assays revealed that copper nanoparticles could be used as a possible raw material for manufacturing medical devices
2. Further in vivo and in vitro studies are needed to confirm the efficacy of copper nanoparticles on hFOB cells. In the future, we hope that copper nanoparticles can be used and applied as a safe and effective modification for implant surface in the treatment and prevention of bacterial infection

## Figures and Tables

**Figure 1:** The optical density of Ti, Ti Cu, Ti HA, and Ti Cu/HA at day 1 and day 3.

**Figure 2:** The cell viability of Ti, Ti Cu, Ti HA, and Ti Cu/HA at day 1 and day 3.

**Figure 3:** The morphology of hFOB cells cultivated with (a) DMEM/F12, (b) Ti, (c) Ti Cu, (d) Ti HA, and (e) Ti Cu/HA extract for one day.

**Figure 4:** The morphology of hFOB cells cultivated with (a) DMEM/F12, (b) Ti, (c) Ti Cu, (d) Ti HA, and (e) Ti Cu/HA extract for three days.

**Figure 5:** The morphology of hFOB cells cultivated with (a) Ti, (b) Ti Cu, (c) Ti HA, and (d) Ti Cu/HA for one day (the arrows showed the cells that attached to coating layer).

**Figure 6:** The morphology of hFOB cells cultivated with (a) Ti, (b) Ti Cu, (c) Ti HA, and (d) Ti Cu/HA extract for three days.

**Table 1:** Comparison of mean differences of the cell viability among treatment groups at day 1and 3.

Time	Comparison		MD	95% CI	*p* value
Day 1	Ti	Ti Cu	6.54	-12.43, 25.52	0.811
		Ti HA	-27.61	-46.58, -8.64	<0.001^∗∗∗^
		Ti Cu/HA	-29.32	-48.29, -10.35	<0.001^∗∗∗^
	Ti Cu	Ti HA	-34.15	-53.13, -15.18	<0.001^∗∗∗^
		Ti Cu/HA	-35.87	-54.84, -16.89	<0.001^∗∗∗^
	Ti HA	Ti Cu/HA	-1.71	-20.68, 17.26	0.996

Day 3	Ti	Ti Cu	-4.75	-23.63, 14.13	0.916
		Ti HA	-37.04	-55.93, -18.16	<0.001^∗∗∗^
		Ti Cu/HA	-44.08	-62.97, -25.21	<0.001^∗∗∗^
	Ti Cu	Ti HA	-32.29	-51.18, -13.41	<0.001^∗∗∗^
		Ti Cu/HA	-39.33	-58.22, -20.45	<0.001^∗∗∗^
	Ti HA	Ti Cu/HA	-7.04	-25.92, 11.84	0.772

^∗∗∗^ = *p* > 0.001.

## Data Availability

All data are available within the manuscript.
